# Untargeted Metabolomic Profiling Using UHPLC-QTOF/MS Reveals Metabolic Alterations Associated with Autism

**DOI:** 10.1155/2020/6105608

**Published:** 2020-09-11

**Authors:** Yujie Liang, Xiaoyin Ke, Zhou Xiao, Ying Zhang, Yangxia Chen, Yingyuan Li, Zhonglei Wang, Ling Lin, Paul Yao, Jianping Lu

**Affiliations:** ^1^Department of Child and Adolescent Psychiatry, Shenzhen Kangning Hospital, Shenzhen Mental Health Center, Shenzhen Key Laboratory for Psychological Healthcare & Shenzhen Institute of Mental Health, Shenzhen, China; ^2^Department of Chemistry, The Chinese University of Hong Kong, Shatin, Hong Kong SAR, China; ^3^Affiliated Shenzhen Clinical College of Psychiatry, Jining Medical University, China; ^4^Department of Medicine, Shenzhen University, Shenzhen, China

## Abstract

Autism spectrum disorder (ASD) is a clinical spectrum of neurodevelopment disorder characterized by deficits in social communication and social interaction along with repetitive/stereotyped behaviors. The current diagnosis for autism relies entirely on clinical evaluation and has many limitations. In this study, we aim to elucidate the potential mechanism behind autism and establish a series of potential biomarkers for diagnosis. Here, we established an ultra-high-performance liquid chromatography-quadrupole time-of-flight mass spectrometry- (UHPLC-QTOF/MS-) based metabonomic approach to discriminate the metabolic modifications between the cohort of autism patients and the healthy subjects. UHPLC-QTOF/MS analysis revealed that 24 of the identified potential biomarkers were primarily involved in amino acid or lipid metabolism and the tryptophan kynurenine pathway. The combination of nicotinamide, anthranilic acid, D-neopterin, and 7,8-dihydroneopterin allows for discrimination between ASD patients and controls, which were validated in an independent autism case-control cohort. The results indicated that UHPLC-QTOF/MS-based metabolomics is capable of rapidly profiling autism metabolites and is a promising technique for the discovery of potential biomarkers related to autism.

## 1. Introduction

Metabolomics, or metabonomics, is one of the developing “-omics” technologies. As a part of the rapidly growing field of postgenomics, which also includes transcriptomics and proteomics, much of the research in metabolomics is aimed at simultaneously characterizing the large numbers of metabolites in biological systems to a pathophysiological intervention or genetic modification. The main methods of metabonomic research are high-throughput chemical analysis and multivariate data analysis. Nuclear magnetic resonance (NMR) and mass spectrometry (MS) fall under the category of high-throughput metabolite profile analysis methods and are the most efficient and widely used [1, 2]. NMR technology allows for simplicity in sample preparation, which enables maintenance of the original nature of the sample. However, there are some drawbacks; until now, NMR has been more suitable for situations that require repeated testing and often results in images with relatively low resolution and sensitivity. On the other hand, MS technology is more sensitive than NMR, enabling metabolites to be detected at picomolar (pmol) concentration levels. Multistage mass spectrometry can be used to accurately obtain the molecular weight of compounds and has been recently combined with ultra-high-performance liquid chromatography (UHPLC), which results in a high level of resolution and sensitivity, and with the development of combined technologies, scientists have combined UHPLC with quadrupole time-of-flight (QTOF) mass spectrometry. This combination, called the UHPLC-QTOF/MS analysis technology, has evolved into the development of sensitive, accurately, and highly reproducible analytical platforms that allow for the determination of hundreds of metabolites in parallel [3–5]. UHPLC-QTOF/MS can be used to analyze lower concentrations of differential metabolites in samples more quickly and comprehensively, making it easier to find potential biomarkers.

The field of metabolomics can also be further divided based on different research purposes into untargeted and targeted metabolomics [6]. Targeted metabolomics focuses on the analysis of specific clusters of metabolites related to certain metabolic pathways, whereas untargeted metabolomics, also known as discovery metabolomics, is a global analysis of different metabolomics between the control group and the experimental group. Metabolomic-based technologies can be used to identify specific biomarkers or conduct metabolic profiling of complex diseases at development and prognosis. Metabolomics has become a promising tool for the research of etiology, biomarker discovery, early diagnosis, and treatment response biomarkers for neuropsychiatric disorders [7]. Previously, metabolomic strategies have been widely used to characterize human metabolic status in the field of central nervous system disorders such as Parkinson's, Alzheimer's, and Huntington's diseases, as well as various neuroinflammatory disorders [8–10]. Metabolomics has also gradually been applied towards the research area of neurodevelopmental disorders including bipolar disorder, autism spectrum disorder (ASD), Rett syndrome (RTT), and schizophrenia [11–14].

Autism spectrum disorders are some of the most common human neuropsychiatric diseases, causing behavioral difficulties and impairment in social interaction. It is estimated that autism affects 1–1.5% of the world population [15]. Diagnosis of autism generally relies on symptom checklists that primarily focus on the person's thoughts and behaviors, thus lacking in precision and repetition. Due to the neurodiversity and heterogeneity of their phenotypic effects, the underlying molecular mechanisms and pathways are still ambiguous. Identification of metabolic biomarkers would assist in their early detection and diagnosis and be beneficial to mechanism studies. To date, numerous studies have utilized metabolomics to profile autism spectrum disorder but have not generated applicable genetic biomarkers for clinical use [16, 17].

In this study, UHPLC-QTOF/MS technology was used to optimize the detection process, chromatography, and mass spectrometry conditions for high-throughput untargeted metabolomic profiling of autism spectrum disorder. A total of 40 autism patients and 40 normal healthy subjects as controls were enrolled, and urine samples were analyzed using the UHPLC-QTOF/MS platform to identify potential metabolite markers associated with autism.

## 2. Methods

### 2.1. Participant Recruitment and Study Design

Clinical autism samples were collected from hospitalized patients in Shenzhen Kangning Hospital, which approved of the study. Urine samples from a total of 40 autism patients and 40 healthy controls were included for UHPLC-QTOF/MS analysis. They were split into two sets: a training set of 60 samples (30 autism and 30 controls) and an independent validation set of 10 ASD and 10 controls.

The selection criteria for autistic participants were set as follows: (i) ASD diagnostic criteria according to the American Psychiatric Association's Diagnostic and Statistical Manual of Mental Disorders (DSM-IV-TR [7]), (ii) children 3-12 years of age, and (iii) exclusion of children with hearing impairments and other neurodevelopmental disorders.

We also excluded individuals with other neurodevelopmental disorders: Rett syndrome, Asperger's syndrome, Fragile X syndrome, disintegrating psychosis (CDD), and other extensive developmental disorders (PDD-NOS). Individuals with major metabolic or genetic diseases were also excluded. Standardized scales, including the Autism Diagnostic Observation Schedule (ADOS), Autism Diagnostic Interview-Revised (ADI-R) and Childhood Autism Rating Scale (CARS), and Autism Behavior Checklist (ABC), were used to assess the severity of each symptom. We also record the clinical symptoms of autistic patients in detail.

The selection criteria for children in the healthy control group were set as follows: (i) children 3-12 years of age and (ii) healthy children with typical development, with exclusion of participants with mental retardation, language impairment, and mental development disorder. Normal healthy controls were confirmed using the normal control criteria of the SCID (Structured Clinical Interview for DSM Diagnosis).

### 2.2. Sample Collection

Each participant was given a standardized dietary recipe, and no other drugs were taken within 2 weeks before collection of samples, which were obtained from each individual at around 8 am after overnight fasting. Immediately after centrifugation, each resulting urine supernatant was aliquoted in a 1.5 mL sterile Eppendorf tube and frozen for storage at -80°C before use.

### 2.3. Chemicals and Reagents

LC-MS grade water, methanol, and acetonitrile were purchased from CNW Technologies (GmbH, Dusseldorf, Germany). High-performance liquid chromatography- (HPLC-) grade ethanol and acetone were obtained from Merck & Co. (Kenilworth, NJ, USA). Ammonium acetate and ammonium hydroxide of LC-MS reagent grade were bought from Sigma-Aldrich (Saint Louis, MO, USA). 2-Chloro-L-phenylalanine was purchased from Shanghai Hengbai Biotech (Shanghai, China).

### 2.4. Metabolite Extraction

Urine samples were thawed on ice at 4°C. 100 *μ*L of sample was taken and placed in 1.5 mL centrifuge tubes before being reconstituted in 300 *μ*L of methanol containing 10 *μ*L internal standard substances. After being vortexed for 3 min and ultrasound treated for 10 min (incubated in ice water), the mixed solution was incubated for 1 h at -20°C to precipitate proteins and then centrifuged at 14,000 rpm at 4°C for 15 min. The supernatant was transferred to a fresh 2 mL LC/MS glass vial, and 20 *μ*L of liquid was taken from each sample to be pooled as QC samples, with 200 *μ*L of supernatant taken for UHPLC-QTOF-MS analysis.

### 2.5. LC-MS/MS Analysis

MS files acquired from the UHPLC system were performed using Agilent 1290 Infinity II with a UPLC BEH Amide column (1.7 *μ*m, 2.1∗100 mm, Waters) coupled to TripleTOF 5600 (QTOF, AB Sciex). The mobile phase consisted of 25 mM NH_4_OAc (ammonium acetate) and 25 mM NH_4_OH (ammonium hydroxide) in water (pH = 9.75) (A), and acetonitrile (B) was carried with an elution gradient as follows: 0 min, 95% B; 7 min, 65% B; 9 min, 40% B; 9.1 min, 95% B; and 12 min, 95% B, which was delivered at 0.5 mL/min. The injection volume included 5 *μ*L of POS (positive polarity) and 2 *μ*L of NEG (negative polarity). A TripleTOF mass spectrometer was used for its ability to acquire MS/MS spectra on an information-dependent basis (IDA) during an LC/MS experiment. In this mode, the acquisition software (Analyst TF 1.7, AB Sciex) continuously evaluates the full-scan survey MS data as it collects and triggers the acquisition of MS/MS spectra depending on preselected criteria. In each cycle, 12 precursor ions with an intensity greater than 100 were chosen for fragmentation at a collision energy (CE) of 30 V (15 MS/MS events with product ion accumulation time of 50 ms each). ESI source conditions were set as follows: ion source gas 1 as 60 psi, ion source gas 2 as 60 psi, curtain gas as 35 psi, source temperature 650°C, and Ion Spray Voltage Floating (ISVF) 5000 V or -4000 V in electrospray ionization in positive (ESI+) ion modes.

### 2.6. Data Processing

ProteoWizard software was used to convert the mass spectrum into mzXML. The preprocessing results generated a data matrix that consisted of the retention time (RT), mass-to-charge ratio (*m*/*z*) values, peak intensity, peak identification, peak extraction, peak integration, and peak alignment. The minfrac was set to 0.5 with a cutoff of 0.6. Additionally, the self-written R package and in-house self-built secondary mass spectrometry database were applied in metabolite identification.

### 2.7. Multivariate Data Analysis

Clustering of QCs was assessed by principal component analysis (PCA) according to total peak area data in order to compare analytical variability with biological variability. The preprocessed data sets were used as input to SIMCA P+ version 14.0 (Umetrics, Umea, Sweden). The training sets of these data sets were tested individually in order to find the best orthogonal partial least squares discriminant analysis (OPLS-DA) model. Model development was performed in order to select a minimum set of predictive metabolites (VIP > 1.5) that were the most implicated in the difference between the ASD and control samples. Logistic analysis with a receiver operating characteristic (ROC) curve was employed for analysis and validation of each biomarker. A combined ROC analysis was performed for panel diagnosis [18, 19]. All tests were considered statistically significant at *P* < 0.05.

## 3. Results

### 3.1. Demographic and Clinical Characteristics of Participants

80 subjects (40 autism and 40 healthy controls) were recruited. Information was collected on each participant, including age, sex, medication, and age at sampling. Diagnosis of ASD was performed using the Autism Behavior Checklist (ABC) and Childhood Autism Rating Scale (CARS). CARS scores were used to measure the behavior characteristic of autism, which consists of 15 domains: listening response, visual response, smell and touch response, nonverbal communication, relating to people, emotional response, imitation, body use, object use, fear or nervousness, verbal communication, activity level, level and reliability of intellectual response, adaptation to change, taste, and general impressions. An individual with a CARS score above 30 is considered to have autism. The enrolled subjects were separated into a training set for discovery biomarkers and an independent test set for validation. The characteristics and group separation of study participants are summarized in Table 1.

### 3.2. Quality Control

Chromatography-mass spectrometry is a very complicated and precise system. During the sample detection process, the results may be affected by objective factors such as humidity, temperature, vibration, and aging of the circuit board, which may lead to signal floating and varying degrees of response. Thus, there is a need for a series of quality control methods for data processing. In theory, quality control (QC) samples are all the same, but there will be errors in the process of substance extraction, detection, and analysis, resulting in some differences between QC samples. Thus, we injected ten QCs to equilibrate the chromatographic system before each analytical batch. The QCs and autism or control samples were analyzed in order to compare the analytical and biological variabilities for each batch. As reflected in the PCA scatter plots, QC samples were densely distributed. From Figures 1(a) and 1(b), we can observe the clustering of QC samples closed to the origin of the PCA scatter plot, which indicates that biological variability exceeds analytical variability, pointing to a very high quality of experimental data. This QC step validates all batch series.

### 3.3. Urine Metabolic Profile

The score plot of orthogonal projection to latent structures (OPLS) discriminates urine profiles of autism patients and normal controls. In Figure 2(a), the *t*[1]*P* represents the predicted principal component score of the first principal component, and the *t*[1]*O* represents the orthogonal principal component obtained. Blue dots and green circles represent the autism and control groups, respectively, thus distinguishing the two groups from one another with all samples above a 95% confidence interval (Hotelling's *T*-squared).

We then validated the OPLS-DA model through permutation tests (number of times *n* = 200) to obtain the *R*^2^ and *Q*^2^ values of the random model. The results of the permutation test on the OPLS-DA model are shown in Figure 2(b). In the figure, the abscissa represents the substitution retention of the substitution test, the ordinate represents the value of *R*^2^ or *Q*^2^, and the green dot represents the *R*^2^ value obtained from the replacement test. The blue square dots represent the *Q*^2^ value obtained from the replacement test. As shown in the figure, the original model *R*^2^ is close to 1, indicating that the model established is consistent with the real situation of the sample data. The *Q*^2^ is close to 1, indicating that if new samples are added to the model, an approximate distribution will be obtained. Permuted *R*^2^ values to the left of the intercept were lower than the original point to the right, and all *Q*^2^ values on the permuted data set to the left are lower than the *Q*^2^ value to the right, indicating that the original model was robust without overfitting.

### 3.4. Predictive Potential of Biomarkers

Differential metabolites that participate in discrimination of the children with autism and healthy controls were selected based on the variable importance in projection (VIP) values and a statistical test for difference (*P* < 0.05) between patients with autism and controls. The 24 metabolites were identified with VIP > 1.5 (Table 2). In order to define the top potential metabolite biomarkers for diagnosis, multiple logistic regression analysis and receiver operating characteristic (ROC) curves were drawn for the training and test sets (Figure 3). Logistic analysis results supported the role of urinary levels of nicotinamide, D-neopterin, anthranilic acid, and 7,8-dihydroneopterin as potential biomarkers that indicate a significant discrimination of autism (Figure 3(a)). We then assessed the diagnostic efficiency of the potential biomarkers using ROC analysis. The areas under the receiver operating characteristic (ROC) curve (AUCs) were 0.912 for nicotinamide, 0.822 for anthranilic acid, 0.840 for D-neopterin, and 0.813 for 7,8-dihydroneopterin, respectively (Figure 3(a)). Furthermore, the diagnostic potential of the 4-metabolite panel was also evaluated. AUCs were 0.891 in the training set and 0.822 in the test set for distinguishing patients with autism from healthy individuals, indicating an excellent clinical diagnosis efficiency for this set of metabolite biomarkers.

## 4. Discussion

Autism usually initiates early in childhood and persists throughout the rest of an individual's life. Autism affects an estimated 13.1 to 29.3 per 1,000 children and is the fastest-growing developmental disability worldwide, rendering it a major public health challenge [20]. Currently, diagnosis of autism is mainly based on clinical interviewing and behavior assessment of characteristics such as impairments in social communication and social interaction, restricted interests, and repetitive behaviors. The lack of objective diagnostic indicators severely restricts the ability to conduct early and rapid diagnosis [21]. Obtaining specific biomarkers through metabolomic research is an important avenue for establishing early screening and diagnostic methods. In recent years, a large number of metabolomic studies have found that autism is accompanied by disturbances in multiple metabolic pathways such as intestinal microbial metabolism, energy metabolism, and oxidative stress [22–24]; thus, metabonomic profiling may be a promising and effective means of identifying variations in metabolite with clinical significance. Additionally, urine from living individuals is a preferable and more accessible biofluid for such screening owing to its noninvasive method of collection and availability in large quantities.

Despite the advancement of ongoing research in the field of metabolomic modeling of autism disorders, there are still many limitations to keep in mind, with the most prominent limitation being detection sensitivity. The most commonly used method of ^1^H NMR spectrometry has a relatively low sensitivity and a limited detection dynamic range, making ^1^H NMR not particularly suitable for analyzing a large number of samples with low metabolite concentrations. With the relatively recent development of time-of-flight (TOF) mass spectrometry and ultra-fast liquid chromatography (UFLC), which have high selectivity and sensitivity, we can now perform quantitative and qualitative analysis of multiple metabolites on samples at the same time [25, 26]. These methods are currently being used as the preferred technology for all aspects of metabolomic research, but to date, there has not been a comprehensive global evaluation of small-molecule metabolites using UHPLC-QTOF/MS in the context of ASD [27].

The first set called the training set was used for a metabolomic discovery analysis of urine to identify metabolites that could be used in discrimination of autism cases and controls. The newly identified metabolites were further validated in an independent validation set of autism cases and controls. In line with this design, we identified four metabolites that allow for good discrimination between the autistic and control subjects, suggesting that these four metabolites could yield the highest predictive power for further diagnostic applications. Each of the potential biomarkers, nicotinamide, anthranilic acid (vitamin L1), D-neopterin, and 7,8-dihydroneopterin, performed well in regard to the area under the curve in analysis (>0.75), and we found that combining a panel of the four parameters can improve diagnostic performance and shows more sensitivity and specificity for discrimination of autism patients from controls. The specificity of the combination of these biochemical biomarkers also helps distinguish probands with autism from the external test set, suggesting that our model has a good predictive ability. However, the specificity of the combination of these biochemical biomarkers regarding other neurodevelopmental disorders should still be evaluated in future studies.

Disruption of the tryptophan kynurenine pathway has been observed in previous research, suggesting that the kynurenine (KYN) pathway is activated in various neuroinflammatory states of ASD [28]. Altered kynurenine pathway metabolites serve as a new potential biological diagnostic marker in a Ptchd1 KO mouse model of human autism spectrum disorders [29]. In our research, we have identified three metabolites, anthranilic acid, 8-dihydroneopterin, and neopterin, which are associated with the tryptophan kynurenine pathway. 8-Dihydroneopterin has been used as an indicator of immune system activation and was the most dazzling inflammatory marker over other traditional biomarkers [30–32]. On the other hand, neopterin is an oxidized form of 7,8-dihydroneopterin, a product of *γ*-interferon-mediated upregulation of GTP cyclohydrolase I (GTPCH1) [33]. Neopterin has been extensively used as a clinical marker of immune activation during inflammation in a wide range of conditions and stressors [34, 35]. Increased inflammation and oxidative stress have been reported in autistic children [36], and it is hypothesized that increased production of inflammatory markers 8-dihydroneopterin and neopterin could play a role in the pathophysiology of autism. Anthranilic acid acts as an intermediate in the biosynthesis of tryptophan, serving as a potential biomarker for other neurodevelopment disorders and as a target for treatment of schizophrenia [37, 38]. Thus, anthranilic acid metabolites are potential diagnostic biomarkers for neurodevelopmental disorders, and the involvement of pathways related to the tryptophan kynurenine pathway suggests that metabolites play an important role in the effects of psychostimulants. The translational perspective, which integrates the study of metabolomics, can shed light on the possible molecular and biological sources of autism.

Recently, a large number of metabolomic studies have revealed that ASD is accompanied with intestinal microbial metabolism, energy metabolism, oxidative stress, and other metabolic pathway disorders, but the fluctuations of some metabolic products involving these pathways have shown controversial results. The unified standardization of the software and databases and different instruments need to be established. Our method could achieve higher resolution, greater sensitivity, and rapid separation, and the UHPLC-QTOF/MS system provides a better opportunity to reveal the most discriminant metabolites for identification of ASD children.

## 5. Conclusion

Our exploratory study has identified several of the metabolites that may be involved in associated biological processes relating to autism spectrum disorder. Our findings serve to shed light on the biomarkers and metabolic mechanism involved in neurodevelopmental disorders such as autism through untargeted UHPLC-QTOF/MS-based urinary metabolomic analysis.

## Figures and Tables

**Figure 1:** PCA scatter plot of quality controls (QCs) and controls injected during each batch analysis. (a) Scatter plot for autism patients and QCs are, respectively, colored with blue dots and red triangles. (b) Scatter plot for controls and QCs are, respectively, colored with green circles and red triangles.

**Figure 2:** (a) OPLS score plot models of autism patients vs. normal controls. *R*^2^*X* = 0.393, *R*^2^*Y* = 0.894. (b) Plot of *R*^2^*Y* and *Q*^2^ from permutation tests in OPLS-DA models.

**Figure 3:** Diagnostic performances of the urinary metabolite parameters in ASD. (a) ROC curve analysis: nicotinamide, anthranilic acid (vitamin L1), D-neopterin, and 7,8-dihydroneopterin as biomarkers of ASD. (b) ROC curve cross-validation based on the combined metabolic biomarker panel could significantly discriminate autism from a healthy individual. AUC: area under the ROC curve; ROC: receiver operating characteristic.

**Table 1:** Descriptive and clinical characteristics of children with autism and healthy control children (TD).

	Training set		Validation set	
Participants	Autism (*N* = 30)	Control (*N* = 30)	Autism (*N* = 10)	Control (*N* = 10)
Gender (male : female)	19 : 11	16 : 14	6 : 4	7 : 3
Age (mean ± SD)	6.5 ± 3.68	6.28 ± 3.25	6.6 ± 2.31	7.08 ± 2.85
ABC total score (mean ± SD)	67.35 ± 14.3	—	56.89 ± 10.6	—
CARS total score (mean ± SD)	34.5 ± 3.9	—	32.1 ± 2.2	—

ABC: Autism Behavior Checklist; CARS: Childhood Autism Rating Scale; SD: standard deviation.

**Table 2:** Differential metabolites for autism and their metabolic pathways.

Metabolite	Ion (*m*/*z*)	Rt	VIP	*P* value	Fold change (autism/control)	Pathway
Nicotinamide	164.0780128	314.4465	2.04	0.03	1.84	Nicotinate and nicotinamide metabolism
Phosphorylcholine	184.0770546	491.186	2.01	0.02	2.34	Phosphorylcholine metabolism
Gly-Glu	205.0852678	401.053	1.74	0.03	1.47	Amino acid metabolism
Acetylcarnitine	226.1098247	202.887	1.85	0.04	2.60	Acetyl-CoA synthase
Ala-Thr	235.0684618	234.5185	2.20	0.02	1.42	Amino acid metabolism
Thr-Asp	235.0948054	405.1215	1.59	0.03	1.39	Amino acid metabolism
His-Pro	235.1210422	143.171	1.58	0.05	1.78	Amino acid metabolism
Bethanechol cation	238.0473387	384.975	2.39	0.01	1.91	Unknown
Pro-Ser	241.0583313	314.282	1.24	0.04	0.66	Amino acid metabolism
D-Neopterin	254.08997	324.551	1.60	0.05	1.71	Tryptophan kynurenine pathway
7,8-Dihydroneopterin	256.1055818	332.338	1.58	0.04	1.84	Tryptophan kynurenine pathway
5-Aminopentanoic acid	257.1511912	194.7525	1.27	0.05	2.94	Catabolism of lysine
Lys-Pro	261.1903229	222.931	1.84	0.02	1.54	Amino acid metabolism
Anthranilic acid (vitamin L1)	275.1038159	282.982	1.68	0.02	2.18	Tryptophan kynurenine pathway
1-Methyladenosine	282.120322	132.113	1.93	0.03	1.50	Modified nucleosides
3′-O-Methylinosine	283.0969971	35.517	1.79	0.02	1.55	Modified nucleosides
Val-Met	290.1604362	308.2965	2.30	0.00	1.81	Amino acid metabolism
S-Methyl-5′-thioadenosine	298.0970956	100.968	1.35	0.04	1.66	Unknown
N-Acetylaspartylglutamate (NAAG)	305.097723	412.4945	1.70	0.02	1.42	Neurotransmitter
1-Naphthol	306.1546719	392.709	1.96	0.00	1.86	Naphthalene metabolites
N-Acetylneuraminic acid	310.1131559	359.178	2.01	0.02	1.83	Sialic acid pathway
Deoxyinosine	313.1065711	35.563	2.11	0.01	1.74	Purine metabolism
Met-Gln	319.1497604	390.399	1.95	0.01	1.39	Amino acid metabolism
Behenic acid	358.365623	38.136	1.56	0.04	1.48	Lipid metabolism

## Data Availability

Data used to support the findings of this study are included within the article.
